The article "Changes in serum and cerebrospinal fluid cytokines in response to non-neurological surgery: an observational study" was published in 2012. Journal: J Neuroinflammation.

# Changes in serum and cerebrospinal fluid cytokines in response to non-neurological surgery: an observational study

**DOI:** 10.1186/1742-2094-9-242

**Published:** 2012-10-24

**Authors:** Sara Bromander, Rolf Anckarsäter, Marianne Kristiansson, Kaj Blennow, Henrik Zetterberg, Henrik Anckarsäter, Caroline E Wass

**Affiliations:** 1 Institute of Neuroscience and Physiology, University of Gothenburg, Gothenburg, Sweden; 2 Department of Anesthesiology and Intensive Care, Kungälv Hospital, Stockholm, Sweden; 3 Department of Clinical Neuroscience, Division of Forensic Psychiatry, Karolinska Institutet, Stockholm, Sweden; 4 Division of Brain and Therapeutics, Department of Psychiatry, University of Toronto and the Schizophrenia Program, Centre for Addiction and Mental Health (CAMH), Toronto, ON, Canada; 5 Institute of Neuroscience and Physiology, Department of Forensic Psychiatry, Gothenburg University, Sahlgrenska Academy, Wallinsgatan 8, 43141, Mölndal, Sweden

**Keywords:** Cytokine, Blood–brain barrier, Central nervous system, Arthroplastic surgery, Cortisol, Albumin, Interleukin, Inflammation

## Abstract

**Background:**

Surgery launches an inflammatory reaction in the body, as seen through increased peripheral levels of cytokines and cortisol. However, less is known about perioperative inflammatory changes in the central nervous system (CNS).

Our aim was to compare inflammatory markers in serum and cerebrospinal fluid (CSF) before and after surgery and evaluate their association with measures of blood–brain barrier (BBB) integrity.

**Methods:**

Thirty-five patients undergoing knee arthroplastic surgery with spinal anesthesia had CSF and serum samples drawn before, after and on the morning following surgery. Cytokines and albumin in serum and CSF and cortisol in CSF were assessed at all three points.

**Results:**

Cytokines and cortisol were significantly increased in serum and CSF after surgery (*P*s <0.01) and CSF increases were greater than in serum. Ten individuals had an increased cytokine response and significantly higher CSF/serum albumin ratios (*P*s <0.01), five of whom had albumin ratios in the pathological range (>11.8). Serum and CSF levels of cytokines were unrelated, but there were strong correlations between CSF IL-2, IL-10 and IL-13, and albumin ratios (*P*s <0.05) following surgery.

**Conclusion:**

Cytokine increases in the CNS were substantially greater than in serum, indicating that the CNS inflammatory system is activated during peripheral surgery and may be regulated separately from that in the peripheral body. CSF cytokine increase may indicate sensitivity to trauma and is linked to BBB macromolecular permeability.

## Introduction

Aseptic trauma, such as peripheral surgery, can lead to an inflammatory response in the central nervous system (CNS), which has been associated with the development of postoperative delirium, depression and cognitive decline [1-3]. Approximately a quarter of geriatric patients undergoing surgery experience postoperative decline in cognitive function, indicating that vulnerable populations is may be at high risk of perioperative insults [4].

The article "Changes in serum and cerebrospinal fluid cytokines in response to non-neurological surgery: an observational study" was published in 2012. Journal: J Neuroinflammation.

Inflammation can be described as the reaction in the body to something adverse, such as trauma or infection. An inflammatory reaction in the brain is increasingly seen as the culprit behind “classical sickness behavior,” often regarded as a model for depression [5]. The old paradigm of an immunologically privileged CNS has been overturned by accumulating evidence showing an intimate relationship between the CNS and the peripheral immune system [6]. Reactions caused by experimental peripheral injection of lipopolysaccharide antigen (LPS), treatment with cytokines to combat illnesses like cancer and hepatitis, as well as surgery have all been shown to have a profound impact on the brain, affecting both mood and cognition [1-3]. Cytokines are a group of important inflammatory mediators [7,8] that act in cascades, inducing or inhibiting each other. Some cytokines, such as interleukin (IL)-1, IL-2, IL-6, and IL-8, and tumor necrosis factor (TNF), generally act in a pro-inflammatory fashion while others, such as IL-4, IL-10 and IL-13 have anti-inflammatory effects, and their intricate balance is crucial for maintaining health [8]. Basal levels of different cytokines and the magnitudes of their increases during inflammation vary between individuals and are under the influence of both different gene variants and environmental factors, e.g. such nutrition [9,10].

Peripherally produced cytokines can enter the brain in several different ways. Some cytokines (for example, TNF) have been shown to cross the blood–brain barrier (BBB) within 30 minutes of intravenous injection [11]. The endothelial cells that make up the BBB may also synthesize cytokines, thus activating an inflammatory process in the brain. Cytokines induced by peripheral inflammation may bind to receptors associated with peripheral afferent nerves (that is, part of the vagus nerve), which, in turn, relay signals to the brain that set off cytokine synthesis [12,13]. In the CNS, cytokines are synthesized both by activated microglia that have migrated as phagocytic cells from the periphery and by microglia, astrocytes and neurons indigenous to the brain [14]. Another well-known and important player in the immune system is the stress hormone cortisol. In its unbound form, cortisol easily passes the BBB [15] and has a profound effect on both CNS and peripheral immune responses [16]. Moreover, levels of cortisol in CSF have also been shown to be associated with delirium after surgery [17]. An orthopedic intervention like knee arthroplasty can be described as trauma under controlled circumstances. Even during spinal blockade, orthopedic surgery is stressful for the whole organism, as illustrated by bradycardia during cementation of protheses [18]. Peripheral surgery sets off an inflammatory reaction in the body, emanating from the surgical wound and manifested as increased levels of inflammatory markers [19,20]. It seems less clear that an inflammatory reaction in the CNS could be elicited, and only a few studies of inflammatory reactions in the CNS elicited by surgery have been published. Levels of cytokines in CSF during an operative intervention have mostly been studied in connection with brain surgery and major heart surgery [21,22]. In 1999, however, Yeager *et al.* found that CSF concentrations of IL-6 increased significantly, while IL-10 remained unchanged after hip surgery [23]. A recent study assessed patients going through an intervention to correct nasal CSF leakage. They were found to have increased levels of CSF S100B, IL-10 and TNF 24 hours following surgery [24]. MacLullich and colleagues [25] found increased CSF IL-8 in patients with postoperative delirium after hip surgery. Thus, while current literature suggests that a peripheral surgical intervention can induce inflammatory reactions in the CNS, further study is needed on the connections between central and peripheral inflammatory responses to surgical stress not directly involving the CNS or the heart. Therefore, in the present study, an array of peripheral and CNS inflammatory markers were assessed in samples from before, three hours after and the day after knee arthroplastic surgery. This is a standardized intervention, which does not involve the CNS or an area of the body that is innervated by the vagus nerve or other afferent cranial nerves, thus avoiding direct immune stimulation of the CNS inflammatory system via this route [26,27]. To investigate the relationship between BBB permeability and inflammatory markers in the brain, serum/CSF albumin ratios [28] were assessed and compared with levels of inflammatory markers.

The article "Changes in serum and cerebrospinal fluid cytokines in response to non-neurological surgery: an observational study" was published in 2012. Journal: J Neuroinflammation.

The aims were:

1. to assess changes in serum and CSF concentrations of cytokines from baseline before non-neurological orthopedic surgery (knee arthroplastics) to three hours post-surgery and the following morning.

2. to assess changes in CSF cortisol concentrations during and after surgery.

3. to investigate the relationship between peripheral and central cytokine levels.

4. to examine the relationship between relative changes in CSF cytokines and cortisol during and after surgery.

## Methods

### Subjects

Thirty-five patients, undergoing knee arthroplastic surgery (20 men, 15 women, aged 51 to 82 years, median age: 73) gave written consent to participate in the study, which was approved by the University of Gothenburg Ethical Review Board. The study protocol has previously been described in detail [29]. Exclusion criteria included the use of anti-Parkinson medication, corticosteroids, antidepressants, antipsychotics and anticoagulant treatment. Seven patients had diabetes mellitus and 21 had hypertension. A previous report on the present sample showed reduced CSF/serum albumin ratios in almost all patients during peripheral surgery [29]. Analysis of baseline CSF/serum albumin ratios identified four patients with abnormal ratios (that is, >11.8). Three hours after surgery, the four individuals with baseline abnormal ratios as well as two additional patients demonstrated CSF/serum albumin ratios >11.8, and three of the patients with abnormal levels at baseline also had abnormal levels the morning following surgery (for a detailed description of these patients see [29]). Since one of the aims of the present study was to investigate relationships between variations in BBB permeability and central inflammatory reactions, the initial analyses included all subjects, regardless of CSF/serum albumin ratios.

### Surgical procedure and sampling

After a subcutaneous local anesthesia with 10 mL 0.5% mepivacaine, a lumbar puncture was performed with an 18-gauge Portex™ (Smiths Group, London, United Kingdom) epidural needle in the L3 to L4 interspace. After discarding about 2 mL of CSF, 12 mL of CSF was sampled and gently mixed before administration of any intrathecal drugs. These baseline CSF samples are referred to as the “A-samples.” Fifteen mL of blood for serum analyses was sampled at the same time. Three hours after completion of the operation, “B-samples” were collected, and on the morning after the intervention, “C-samples” were drawn by the same routine to avoid any admixture of puncture bleeding or ongoing infusions. CSF and serum samples were centrifuged at 2,000 g for 10 minutes to separate cells and other insoluble material from the aliquots, and pipetted in new tubes for transport to the neurochemistry laboratory. Aliquots were stored at −80° C until biochemical analyses were performed. All subjects had fasted at least six hours before surgery. Any glucose infusions and pharmacological agents administered during and after surgery were carefully registered. As the spinal blockade was still active after surgery, the patients remained fasting when the second CSF sampling was performed, but were free to eat in the evening after the operation. During surgery, propofol was administered as a continuous infusion to all patients, using the bispectral index (BIS) to titrate the dosage for an optimal sedation of BIS 70 (for a detailed description of medications and dosages, see Anckarsater *et al.*, 2007). No complications except pain breakthrough were noted during the study.

The article "Changes in serum and cerebrospinal fluid cytokines in response to non-neurological surgery: an observational study" was published in 2012. Journal: J Neuroinflammation.

### Neurochemical analysis

Cytokines were analyzed using the Human TH1/TH2 10-Plex Assay Ultra-Sensitive Kit as described by the manufacturer (Meso Scale Discovery, Gaithersburg, MD, USA). This kit includes analyses of IL-1β, IL-2, IL-4, IL-5, IL-8, IL-10, IL-12, IL-13, IFN-γ and TNF. The lowest level of detection was 0.61 pg/mL. Serum and CSF albumin concentrations were determined by nephelometry on the Beckman Coulter IMMAGE® (Beckman Coulter, Pasadena, CA, USA). The albumin ratio was calculated as CSF albumin (mg/L)/serum albumin (g/L) [28]. Cortisol concentration in CSF was determined by radioimmunoassay using the Spectria CORTISOL (125I) kit (Orion Diagnostica, Sollentuna, Sweden). Intra-assay coefficients of variation were below 10% for all analyses.

### Statistical methods

All statistical analyses were performed using the SPSS 18.0 software (International Business Machines Corporation, Amonk, New York, USA). As the distribution of cytokine levels was skewed due to the lower detection level of the analysis kit (0.61 pmol/mL), nonparametric methods were used. For comparing the cytokine levels at A, B and C, Friedman’s repeated measures analysis of variance by ranks, followed by Wilcxon Signed Rank test for *post hoc* comparisons between pairs were used. To analyze the relationship between peripheral and central levels of cytokines, cortisol and CSF/serum albumin ratios (in absolute levels), and the relationship between peripheral and central fluctuations in cytokines (relative change in cytokine levels was computed as concentration at C divided by concentration at B, B divided by A, and C divided by A), Spearman correlations were computed. For analysis of differences in CSF/serum albumin ratios and cytokine levels between subgroups, Mann–Whitney U-tests were used. All tests were two-tailed, and significance levels were set at 0.05.

## Results

### Serum and CSF cytokine levels were increased following peripheral surgery

#### Serum

Repeated measures analyses identified significantly increased serum concentrations of IL-8 and IL-10 three hours after surgery (at B) and on the morning following surgery (at C). Serum TNF decreased significantly between the A and C samplings (for mean concentrations, standard deviations and statistics, see Table 1). As the changes in serum cytokines were moderate and expected during surgery, they were not further explored.

The article "Changes in serum and cerebrospinal fluid cytokines in response to non-neurological surgery: an observational study" was published in 2012. Journal: J Neuroinflammation.

**Table 1:** Serum and CSF mean (± SD) concentrations (pg/mL) of cytokines at A, B and C

**Serum**	**IFN-γ**	**IL-1β**	**IL-2**	**IL-4**	**IL-5**	**IL-8**	**IL-10**	**IL-12**	**IL-13**	**TNF**
**A**	1.36 ± 1.12 N = 34	0.63 ± 0.06 N = 34	1.20 ± 1.51 N = 34	0.62 ± 0.04 N = 34	1.05 ± 0.91 N = 34	23.98 ± 116.12 N = 34	3.53 ± 4.09 N = 34	3.35 ± 5.02 N = 34	11.81 ± 26.15 N = 34	8.62 ± 3.05 N = 34
**B**	1.49 ± 1.18 N = 34	0.64 ± 0.12 N = 34	0.95 ± 0.64 N = 34	0.62 ± 0.08 N = 34	1.00 ± 0.08 N = 34	26.86 ± 123.50 N = 34	6.00 ± 7.43 N = 34	3.35 ± 5.10 N = 34	10.96 ± 23.36 N = 34	9.35 ± 3.71 N = 34
**C**	1.07 ± 0.78 N = 34	0.64 ± 0.12 N = 34	1.16 ± 1.64 N = 34	0.63 ± 0.10 N = 34	1.61 ± 1.51 N = 34	30.19 ± 126.82 N = 34	9.62 ± 7.28 N = 34	3.11 ± 4.60 N = 34	9.54 ± 19.15 N = 34	7.91 ± 2.25 N = 34
**Friedman′s statistics**	χ2 (2) = 5.009 n.s.	χ2 (2) = 0.857 n.s.	χ2 (2) = 0.364 n.s.	χ2 (2) = 0.286 n.s.	χ2 (2) = 7.013 ***P*** = 0.03*	χ2 (2) = 43.304 ***P*** <0.001***	χ2 (2) = 49.259 ***P*** <0.001***	χ2 (2) = 0.505 n.s.	χ2 (2) = 4.047 n.s.	χ2 (2) = 9.450 ***P*** = 0.009**
**Wilcoxon signed rank test*P*-values**					AB n.s. AC*P*= 0.03* BC*P*= 0.02*	AB*P*<0.001*** AC*P*<0.001*** BC n.s.	AB*P*<0.001** AC*P*<0.001*** BC*P*<0.001***			AB n.s. AC *P*= 0.03* BC n.s.
**CSF**	**IFN-γ**	**IL-1β**	**IL-2**	**IL-4**	**IL-5**	**IL-8**	**IL-10**	**IL-12**	**IL-13**	**TNF**
**A**	0.70 ± 0.29 N = 26	0.63 ± 0.10 N = 25	0.63 ± 0.54 N = 25	0.61 ± 0.00 N = 25	0.61 ± 0.00 N = 25	30.40 ± 8.80 N = 25	0.76 ± 0.22 N = 25	0.64 ± 0.13 N = 25	0.61 ± 0.00 N = 25	0.67 ± 0.14 N = 25
**B**	1.08 ± 0.97 N = 26	0.84 ± 0.47 N = 25	4.74 ± 10.77 N = 25	0.62 ± 0.05 N = 25	1.31 ± 1.87 N = 25	880.68 ± 1975.95 N = 25	6.91 ± 14.69 N = 25	1.54 ± 2.55 N = 25	3.02 ± 5.64 N = 25	2.76 ± 5.07 N = 25
**C**	0.93 ± 0.80 N = 26	0.79 ± 0.35 N = 25	3.38 ± 6.33 N = 25	0.61 ± 0.00 N = 25	0.99 ± 0.79 N = 25	543.20 ± 964.20 N = 25	5.15 ± 9.23 N = 25	1.21 ± 1.91 N = 25	3.26 ± 4.36 N = 25	1.77 ± 2.32 N = 25
**Friedman′s statistics**	χ2(2) = 3.150 n.s.	χ2(2) = 4.839 n.s.	χ2(2) = 19.316 ***P*** <0.001***	χ2 (2) = 4.00 n.s.	χ2 (2) = 10.042 ***P*** = 0.007**	χ2 (2) = 38.000 ***P*** <0.001***	χ2 (2) = 27.758 ***P*** <0.001***	χ2 (2) = 5.892 n.s.	χ2 (2) = 23.343 ***P*** <0.001***	χ2 (2) = 17.956 ***P*** <0.001***
**Wilcoxon signed rank test*P*-values**			AB ***P*** = 0.001*** AC ***P*** <0.001*** BC n.s.		AB n.s. AC ***P*** = 0.002 ** BC n.s.	AB ***P*** <0.001*** AC ***P*** <0.001*** BC n.s.	AB ***P*** <0.001*** AC ***P*** <0.001*** BC n.s.		AB ***P*** <0.001*** AC ***P*** = 0.001*** BC n.s.	AB ***P*** <0.001*** AC ***P*** <0.001*** BC n.s.

The article "Changes in serum and cerebrospinal fluid cytokines in response to non-neurological surgery: an observational study" was published in 2012. Journal: J Neuroinflammation.

#### CSF

In the CSF, concentrations of several cytokines (IL-2, IL-5, IL-8, IL-10, IL-13 and TNF) increased significantly during and after surgery (Table 1), with large effect sizes (IL-2, IL-8, IL-10 and IL-13 all increased to about 500% or more of their initial concentrations, while TNF more than doubled). Relative changes in all of these CSF cytokines showed highly significant intercorrelations (rhos ranging from 0.434 to 0.902 and *P*s from <0.001 to 0.015), indicating that subjects with high increases in one cytokine also had increases in other cytokines.

#### Subgroups with different patterns of CSF cytokine response

As illustrated by the large standard deviations, CSF concentrations of IL-2, IL-10, IL-12 and IL-13 displayed large interindividual variations following surgery, while IL-8 and TNF had more consistent changes. Based on the plotted distributions of the CSF cytokine concentrations, a set of 10 outliers (referred to as “high cytokine responders” (see Figure 1) had substantially higher concentrations than the rest of the sample. This was defined as having either CSF IL-2 >4 pg/mL (individuals coded as e, i, l, m and z), IL-10 >5 pg/mL (individuals coded as a, b, e, f, i, l, m and z), IL-12 >7 pg/mL (individuals coded as e, i and m) or IL-13 >6 pg/mL (individuals coded e, i, j, m, p, y and z) at B and/or C. First, both serum and CSF cytokine concentrations were compared between this group and the rest of the study group to assess whether they were significantly different in their overall cytokine responses. The high responders had significantly higher CSF concentrations of almost all cytokines assessed (IL-2, 4, 5, 8, 10, 12, 13, TNF and INF-γ) at B and C, as well as significantly higher serum concentrations of IL-4 at A and IL-8 at A and B (for mean ranks and statistics, see Table 2).

**Figure 1:** Correlations between CSF/albumin ratios and CSF cytokine levels.

**Table 2:** Differences in CSF and serum cytokine levels between high and low cytokine responders at A, B and C

	**Group**	**csf IL-2**	**csf IL-4**	**csf IL-5**	**csf IL-8**	**csf IL-10**	**csf IL-12**	**csf IL-13**	**csf TNF**	**csf INFγ**	**serum IL-4**	**serum IL-8**
**A**	high responders										19.30 (10)	22.65 (10)
	rest of sample										16.00 (23)	14.54 (23)
	***U,****P****-value***	**n.s.**	**n.s.**	**n.s.**		**n.s.**					92.00, 0.027*	58.50, 0.027*
**B**	high responders	22.80 (10)	18.10 (10)	19.70 (10)	24.30 (10)	22.70 (10)	23.10 (10)	19.50, 0.001	23.80 (10)	21.50 (10)		23.15 (10)
	rest of sample	13.64 (22)	15.00 (21)	14.24 (21)	12.05 (21)	12.81 (21)	12.62 (21)	11.76 (21)	12.29 (22)	14.23 (22)		14.33 (23)
	***U,****P****-value***	47.00, 0.008**	84.00, 0.037*	68.00, 0.042*	22.00, <0.001***	38.00, 0.005**	34.00, <0.001***	16.00, <0.001***	27.00, 0.001***	60.00, 0.016*	**n.s.**	53.50, 0.016*
**C**	high responders	24.00 (10)		25.00 (10)	25.15 (10)	25.00 (10)	23.35 (10)	25.55 (10)		20.65 (10)		
	rest of sample	13.09 (22)		12.64 (22)	12.57 (22)	12.64 (22)	13.39 (22)	12.39 (22)		14.61 (22)		
	***U,****P****-value***	35.00, 0.002*	**n.s.**	25.00, <0.001***	23.50, <0.001***	25.00, 0.001***	41.50, 0.001***		**n.s.**	**68.50, 0.027**	**n.s.**	**n.s.**

Differences between groups based on ranks, with mean rank in cytokine levels and number of patients (n) in the different groups for each cytokine is presented, followed by Mann–Whitney U statistics U-values, *P*-values. The α-level was set to 0.005, *<0.05, ** <0.01, *** ≤0.001.

The article "Changes in serum and cerebrospinal fluid cytokines in response to non-neurological surgery: an observational study" was published in 2012. Journal: J Neuroinflammation.

#### CSF cytokine levels and possible confounding factors

The high cytokine responders also had significantly higher CSF/serum albumin ratios at B (U = 38.00, *P* = 0.003) and C (U = 45.00, *P* = 0.008). Half of these high responders had abnormal albumin ratios (>11.8 as the upper range of the established reference interval for the method) at one or several of the assessment points, while the remaining five subjects had relatively stable albumin ratios within the normal range (Figure 2). CSF cytokine responses were plotted in relationship to albumin ratios. These two factors were significantly correlated for several of the cytokines in the full sample (Figure 1).

**Figure 2:** Albumin ratios at A, B, and C in high cytokine responders (n=10).

To rule out the possibility that the overall increases in CSF cytokines were due to the patients with abnormal albumin ratios (that is, >11.8), these individuals were tentatively excluded from the basic analyses. This exclusion did not markedly alter the serum or CSF cytokine concentrations following surgery, with the exception of serum IL-5, which was no longer significant after the correction for albumin ratios. Since exclusion of individuals with abnormal albumin ratios did not markedly change the pattern of cytokine response following surgery, all individuals, regardless of albumin ratios, were included in the following analyses, except when otherwise stated.

Other potential confounding factors, age, gender, and body mass index (BMI) were evaluated by computing correlation analyses with serum and CSF cytokine concentrations at A, B and C. BMI was negatively correlated with the CSF concentration of IL-8 at baseline (rho = −0.408, *P* = 0.034) and age correlated significantly with serum IL-10 at B (rho = 0.540, *P* = 0.001). No other associations were found.

The article "Changes in serum and cerebrospinal fluid cytokines in response to non-neurological surgery: an observational study" was published in 2012. Journal: J Neuroinflammation.

### CSF cortisol concentrations increased significantly following surgery

Repeated measure analyses identified significant increases in mean CSF cortisol concentrations between A, B and C (χ^2^ (2) = 28.08, *P* <0.001) and pairwise *post-hoc* comparisons revealed the following changes from A (20.61 ± 6.73 nmol/L) to C (51.69 ± 22.24 nmol/L; Z = −4.41, *P* <0.001) and from B (22.05 ± 14.41 nmol/L) to C (Z = −4.49, *P* <0.001) in the whole sample. Exclusion of individuals with albumin ratios above 11.8 did not markedly affect these results (χ^2^ (2) = 21.09, *P* <0.001) and no correlations between albumin ratios and CSF cortisol concentrations were detected at any of the assessment points.

#### Confounders

To control for the time of sampling, age, BMI and gender, correlation analyses with CSF cortisol levels were computed. Correlations were found between age and cortisol concentrations at A (rho = 0.494, *P* = 0.010) and C (rho = 0.663, *P* <0.001), such that older age was associated with higher levels of CSF cortisol. No other correlations were found.

### No correlation between peripheral and central cytokine levels

To investigate the relationship between peripheral and central levels of cytokines, correlational analysis between CSF and serum levels for each of the cytokines IL-2, IL-5, IL-8, IL-10, IL-13 and TNF were computed. These cytokines were included in the analysis as they significantly changed following surgery, as described above. No significant correlations between serum and CSF concentrations (absolute values) at any sampling were detected.

### Correlations between CSF cytokines and cortisol levels

To investigate whether the various inflammatory markers were intercorrelated, correlations between CSF concentrations of cytokines and cortisol were assessed at A, B and C. CSF cortisol concentrations correlated significantly with CSF IL-10 and IL-8 (rho = 0.422, *P* = 0.025 and rho = 0.386, *P* = 0.043, respectively) three hours after surgery (at B). Relative change in CSF cortisol from three hours after surgery (at the B sampling) to the morning after surgery (at the C sampling) correlated significantly with relative changes in CSF IL-2 (rho = 0.399, *P* = 0.039). However, no other correlations between cortisol and the different cytokines were identified at any of the assessment points.

## Discussion

This naturalistic study indicates that an orthopedic intervention induced significant increases in inflammatory markers, both in the peripheral circulation and the CNS. Remarkably, the cytokines increased with greater magnitude in the CSF than in the serum, and correlations between changes in different CSF cytokines were evident. In addition, cortisol levels in CSF increased significantly following surgery. Subgroup analysis of the cytokine response identified 10 individuals who displayed a larger cytokine response than the rest of the sample following surgery. Half of these individuals also displayed abnormally high CSF/serum albumin ratios. Moreover, serum and CSF concentrations of cytokines did not correlate. However, CSF cytokine levels did correlate significantly with albumin ratios following surgery. A detailed discussion of these results follows below.

The article "Changes in serum and cerebrospinal fluid cytokines in response to non-neurological surgery: an observational study" was published in 2012. Journal: J Neuroinflammation.

### Widespread, markedly increased CSF cytokine levels following surgery: specific cytokine responses and their potential roles

Remarkably, CSF concentrations of both pro- (TNF, IL-2, IL-8) and anti-inflammatory (IL-10, IL-13) mediators were significantly increased postoperatively while, in serum, only IL-8, IL-10 and TNF were affected by surgery. Changes in the CSF concentration of one cytokine were strongly correlated with changes in other cytokines, indicating a unified and widespread pro- and anti-inflammatory response, as expected. Ten individuals were found to display high albumin ratios as well as an exceptionally high CSF cytokine response. Despite not being significantly different from the low responders in CSF cytokine levels before surgery, these individuals displayed significantly and highly enhanced levels of several CSF cytokines. This may indicate that there are individuals without any identified, clinically relevant, neurological or psychiatric disorder that show remarkably heightened neuroinflammatory response to non-neurological surgery. Unfortunately, no psychiatric or neurological assessments following surgery were done in the present study to evaluate whether these individuals were at higher risk for developing postoperative delirium.

The length of the observed reaction in the CSF, which lasted at least until the morning following surgery, may be a reflection of the relatively advanced age of the study population, as the inflammatory reaction is known to be prolonged and increased in old age [30]. Correlational analysis between CSF cytokine levels at C and age did not identify any such correlations; however, this may be due to the restricted age span of the present sample.

Moreover, IL-2 showed an elevation in both CSF and serum following peripheral surgery. IL-2 is a pro-inflammatory cytokine known to enhance dopaminergic transmission. It serves as a neuromodulatory molecule in the CNS, stimulating the HPA-axis and neuronal survival [31], which may explain why there was a significant correlation between CSF IL-2 levels and cortisol following the surgical intervention.

The article "Changes in serum and cerebrospinal fluid cytokines in response to non-neurological surgery: an observational study" was published in 2012. Journal: J Neuroinflammation.

CSF IL-8 levels were markedly increased following surgery, while the peripheral levels were more modestly elevated and returned to normal on the morning after surgery. A variety of cells, including astrocytes activated by IL-1 and TNF, can produce IL-8, which is an important part of the acute phase reaction [32]. IL-8 may contribute to the psychiatric complications of surgery, as it is increased in the CSF of hip fracture patients with postoperative delirium, compared to patients without delirium [25]. It is noteworthy that CSF levels of IL-8 increased by 2,360% from A to B, and by 1,530% from A to C, while in serum the magnitudes of the increases were 11% from A to B and 26% from A to C. The strong increase in pro-inflammatory cytokines is not surprising, as surgery constitutes a significant trauma to the organism. IL-8 may be synthesized in the CSF as well as transported across the BBB, maybe indicated by the correlations between the CSF/albumin ratio and IL-8 at B and C.

Levels of TNF are known to rise early in connection with surgery, and TNF is known to have a very short half-life in serum. It is suspected to play an important role in postoperative cognitive decline [33]. Several studies have shown a sustained generation of TNF in the CNS after peripherally induced inflammation [34-36]. In the present study, levels of TNF increased, both in serum and in CSF, directly after surgery, but then decreased overnight in serum. This would be consistent with earlier studies regarding prolonged increased levels of TNF in the CNS. As TNF has been implicated as playing an important role in conditions like delirium and Alzheimer’s disease, individuals showing a prolonged elevation of TNF in the CNS may be at risk of developing such complications [37].

IL-10 and IL-13 are known mainly as anti-inflammatory cytokines [7]. The increase of IL-10 in CSF, especially after surgery, seems logical, as one of its roles is to down-regulate the immune reaction [38]. IL-13 has been shown to play a neuroprotective role in both animal and human studies [39,40]. This cytokine, as observed in the present sample, would also be expected to increase in response to an inflammatory process.

The mean concentrations of serum IL-4 at all assessment points, and baseline CSF IL-5 and IL-13, were at the lower detection level of the assay. Thus, the assessment of these cytokines may not represent their true concentrations and therefore limits the interpretation of these data.

### CSF cortisol levels increased following surgery but not associated with BBB permeability

Cerebrospinal fluid cortisol changed during surgery, with the most pronounced increase on the morning following surgery. Cortisol excretion follows diurnal endogenous endocrine variations in addition to fluctuations due to external stimuli, such as stress [16]. Some studies suggest that CNS levels of cortisol follow the same diurnal fluctuations as in the periphery; thus it is not possible to say with certainty that the changes seen in this study do not reflect normal fluctuations. The impact of surgical stress on diurnal variations in cortisol levels is insufficiently studied; however, other kinds of stress (for example, depressive illness) are known to blunt these fluctuations [41]. Serum levels of cortisol were not measured in the present study as they are pulsatile and, therefore, unreliable. No correlations between BBB permeability as assessed by albumin ratio and CSF cortisol were found, suggesting that the increase in cortisol may be due to an increase in CNS cortisol levels.

The article "Changes in serum and cerebrospinal fluid cytokines in response to non-neurological surgery: an observational study" was published in 2012. Journal: J Neuroinflammation.

### Cytokine increase and relationship to BBB permeability

CSF and serum concentrations of the various cytokines were not shown to be correlated. However, the relationship between BBB permeability and intrathecal cytokine levels was evaluated to investigate whether the central cytokine increase might be due to disruption in the BBB. Correlations between CSF IL-2, IL-10, IL-13 and BBB permeability, as measured by the CSF/serum albumin ratio, were detected post-operatively in a subgroup of individuals. Specifically, the 10 individuals who displayed exceptionally high CSF inflammatory responses to surgery also had significantly higher albumin ratios compared to those individuals with less pronounced cytokine increases. Five of the subjects displayed abnormally high albumin ratios. No other specific factor that may have contributed to the high cytokine response was detected. The response of IL-2 and IL-13 was most strongly pronounced on the morning following surgery (that is, at C), and there were highly elevated levels of several of the cytokines at B and C. The correlations between IL-2, IL-10, IL-13 at B, IL-10 at C, and albumin ratios, were present but not as strong as in the full sample, indicating that these effects may reflect a normal association between BBB permeability and cytokine response.

Animal studies demonstrate that increased BBB permeability following surgery enables phagocytic cell migration into the brain, where these cells then act as microglia, and consequently increase IL-10 release in the hippocampus [42]. Despite the overlap between the different types of markers (that is, IL-8, IL-10 and TNF) fluctuating in both the CNS and the periphery independent of BBB integrity as assessed by albumin ratio, these results indicate that the intrathecal and peripheral inflammatory systems may be separately regulated in response to surgical trauma. Consequently, it is possible that the increased CNS inflammatory response may be induced via another mechanism than that of increased BBB permeability and the migration of phagocytic cells into the CNS. Furthermore, it cannot be excluded that the turnover of cytokines in the CNS after the intervention is slower than in the periphery, and that this might explain the differences in changes in cytokine levels observed in this study. Prolonged inflammatory reactions in the CNS have been associated with old age [30].

The article "Changes in serum and cerebrospinal fluid cytokines in response to non-neurological surgery: an observational study" was published in 2012. Journal: J Neuroinflammation.

### Limitations

Although there are important limitations to the present study, it should be noted that the study is naturalistic and reflects a true clinical sample. The study sample was small and the participants were older and heterogeneous regarding long-term use of medications and concomitant medical disorders. These confounding variables are inevitable, as knee prosthesis surgery is generally performed on older people. It should be noted that levels of several inflammatory markers increase with age [43,44]. Nineteen of the patients were overweight, with a BMI over 25, and seven had diabetes mellitus, both conditions characterized by increased inflammatory activation [45,46]. Propofol was administered to all patients as anesthesia and has been reported to have anti-inflammatory properties [47,48]. Unfortunately, we cannot rule out other medications taken by the patients having effects on their inflammatory responses [49].

IL-6 is a pro-inflammatory cytokine, which has been extensively studied in connection with cognition and psychiatric states in recent years [50,51]. Due to limitations of the analysis kit, which was chosen for its suitability for CSF analysis, this cytokine was not included in our study. Also, no genetic testing was done, thus it was not possible to determine whether any of the subjects had polymorphisms in any genes known to affect their inflammatory response [52]. For example, apolipoprotein E is a polymorphic lipid transporter protein with multiple biological properties [53]. The ApoE E4 polymorphism of the gene coding for this protein has been associated with increased risk of Alzheimer′s disease [54], and also of postoperative delirium [55]. Individuals carrying this polymorphism seem to have an increased inflammatory reaction to surgery [52]. It cannot be ruled out that those cytokines that had mean concentration detected at the lower detection levels of the assays used may in fact fluctuate in response to the surgical intervention, as their true concentration levels may not have been detected in this study.

As we were unable to have continuous CSF samplings, we chose to collect samples three hours after termination of the intervention to be able to pinpoint chemical reactions during the operation (considering absorption time for CSF [56]). The sampling on the morning after surgery was performed in order to assess the continued inflammatory reaction during the night. Continuing samplings for a longer period was not regarded as feasible, as the patients no longer had any need for intrathecal catheters. We also cannot rule out an inflammatory effect of the catheter or lumbar puncture; this, however, would be a problem in all studies of CSF, and it would be unlikely given the magnitude of changes. As the catheter was made from an inert material and all lumbar punctures were performed by an experienced anesthesiologist, we hypothesize that the inflammatory changes caused by this procedure would be minimal. Confounding by factors affecting the majority of all subjects cannot be eliminated, as the study design did not include a control group. The study includes no formal testing of causation and should be regarded as descriptive on the basis of correlations and observations.

The article "Changes in serum and cerebrospinal fluid cytokines in response to non-neurological surgery: an observational study" was published in 2012. Journal: J Neuroinflammation.

## Conclusion

This is the first study demonstrating a pronounced inflammatory reaction centrally (as reflected in CSF) as a consequence of arthroplastic knee surgery in humans. Notably, the relative cytokine increase in CSF is much larger than in serum. The lack of correlations between peripheral (that is, serum) and central levels of cytokines may indicate that inflammatory reactions in the brain during non-neurological surgery are regulated separately from the periphery. However, a subgroup of subjects revealed a stronger inflammatory response. This effect seemed related to high BBB permeability, suggesting that some individuals, without any known neurological or psychiatric diagnosis, may have a more sensitive BBB and be particularly prone to exaggerated neuroinflammatory responses following peripheral surgery. Considering that CNS inflammation is a risk factor for neuropsychiatric complications, such as postoperative delirium, such individuals may be considered high-risk and may benefit from anti-inflammatory interventions. Consequently, novel approaches for preventing neuropsychiatric surgical complications could possibly target the inflammatory process.

## Abbreviations

BBB: blood–brain barrier; BIS: bispectral index; BMI: body mass index; CNS: central nervous system; CSF: cerebrospinal fluid; HPA-axis: hypothalamic-pituitary-adrenal axis; IL: interleukin; TNF: tumor necrosis factor.

## Competing interests

The authors declare that they have no competing interests.

## Authors’ contributions

SB performed the statistical analysis and prepared the draft of the manuscript. CW also took part in the statistical analysis and draft preparation, and acted as supervisor for SB. HA conceived of the study, participated in its design and coordination and helped to draft the manuscript. RA participated in the design of the study and the recruitment of subjects and performed the actual samplings. HZ and KB participated in the design of the study and performed the laboratory analyses. MK participated in the study design and took part in the preparation of the draft. All authors read and approved the final manuscript.
